# Effects of the Addition of Nb and V on the Microstructural Evolution and Hydrogen Embrittlement Resistance of High Strength Martensitic Steels

**DOI:** 10.1155/2022/4040800

**Published:** 2022-02-24

**Authors:** Bo Liu, Xiaolin Liao, Yuanshou Tang, Yu Si, Yi Feng, Pengjun Cao, Qingwei Dai, Kejian Li

**Affiliations:** ^1^State Key Laboratory of Vehicle NVH and Safety Technology, Chongqing 401122, China; ^2^University of Science and Technology Beijing, School of Mechanical Engineering, Beijing 100083, China; ^3^Chongqing Changan Automobile Co., Ltd., Chongqing 400023, China; ^4^School of Metallurgy and Materials Engineering, Chongqing University of Science & Technology, Chongqing 401331, China; ^5^China Automotive Engineering Research Institute Co., Ltd., Chongqing 401122, China

## Abstract

Hydrogen embrittlement can easily occur in high strength martensitic steel, manifesting itself as a sudden failure or fracture without warning and greatly threatening the safety of automotive applications. Optimizing the composition of the alloy can be performed by matching heat treatment processing methods and controlling the precipitation amounts to form hydrogen traps. In doing so, the hydrogen embrittlement susceptibility of steel can be effectively delayed, reducing the risk of hydrogen-induced delayed cracking. In this study, four kinds of 1500 MPa strength grade martensitic steel were selected for testing and supplemented with different loadings of Nb and V, respectively. Their grains, phases, and precipitations were compared by optical microscopy (OM), electron backscattered diffraction (ESBD), and transmission electron microscopy (TEM) analyses. After the addition of Nb and V, the microstructure was refined, the residual austenite content increased, and the hydrogen embrittlement resistance was significantly improved.

## 1. Introduction

High strength martensitic steels exhibit excellent mechanical properties, which enables them to be extensively applied in the automotive industry [1]. More than 50% of the materials used in the automotive industry consist of steels, and the development of high-performance materials is the key to improving safety performance and industrial competitiveness. Advanced high strength steel has both high strength and good formability, especially a high work hardening index, which helps to improve the energy absorption in the collision process, lightweights the vehicle, and ensures safety. Among the materials with over 1500 MPa strength, hot-formed or cold-formed martensitic steels are the most economical choices [2–5]. However, in using these types of martensitic steels, a major challenge is hydrogen-induced delayed fracture. Traditional ways of improving the performance of martensitic steel include increasing the carbon content, alloying elements, and cyclic quenching, which make the steel more expensive and decrease weld ability. Controlled rolling and cooling with microalloying can effectively improve the performance and economics of the material [6–8].

Nagao et al. studied the fractures of hydrogen-induced cracking of martensitic steel and found that the slip band intersected with the prior austenite grain boundary (PAGB) and ML (ML) boundary. The hydrogen was enriched at the above two interfaces under the action of dislocation transmission, leading to grain boundary and quasicleavage [9]. The high susceptibility of hydrogen-induced delayed fracture of hot-formed steel can be attributed to two aspects. The first aspect is the high dislocation density. Higher dislocation density results in numerous dislocation cell tangles being formed in the matrix, where the dislocation entanglement area is the high-defect area, and the dense network of the dislocation entanglement area can become a facile channel for hydrogen diffusion [10–13]. The second aspect is high residual stress after forming and quenching, which, together with external stress, intensifies the promoting effect of hydrogen diffusion. If hydrogen aggregates toward the higher-stress concentration area, it further increases the risk of hydrogen-induced cracking [14–16]. However, dislocation and stress are difficult to avoid during material preparation. It is well known that adding microalloying elements can reduce hydrogen-induced delayed fracture to improve their residual austenite (RA) and material microstructure and create more hydrogen traps.

Controlling the precipitation of C or N nanocompounds to form a benign “hydrogen trap” in high strength martensitic steel can effectively reduce the risk of hydrogen-delayed cracking [17]. A hydrogen trap can be caused by various microstructural defects, such as PAGB, lath boundaries, high-density dislocations, and interfaces between the second phase particles and matrix. Generally, all steel defects can be used as hydrogen traps. The key to determining the hydrogen trapping ability of defects is to determine the binding energy between defects and hydrogen. A binding energy of ≥50 kJ/mol is a strong trap, while a binding energy of ≤30 kJ/mol is a weak trap [18–22]. The order of all defects according to binding energy is lattice gap < grain boundary < dislocation < vacancy < carbide [23]. A large number of grain boundaries can promote defect homogenization and stress distribution and increase the hydrogen diffusion path distance, thereby realizing hydrogen distribution dispersion in the matrix. Therefore, the high-density grain boundary improves the influence of hydrogen to prevent an excessively high concentration of hydrogen [24–26].

Carbides have the strongest hydrogen trapping ability, and Nagao pointed out that nanoscale (Ti, Mo) C in martensitic steel is more capable of trapping hydrogen than larger particles [27–31]. The decrease in the size and quantity of carbides leads to an increase in the diffusion distance of hydrogen in steel, which is known method used to reduce the susceptibility of hydrogen-delayed fracture in high strength steel.

In recent years, high strength martensitic steels were prepared with the addition of Nb, V, Ti, and Cu elements with different heat treatment processes. Finally, many precipitation forms and their hydrogen trapping mechanisms were studied [23, 32–38]. However, the microstructural refinement of ultra-high strength steels has been less reported. In this study, Nb and V were added to high strength steel, and their grain sizes, boundaries, and RA contents were compared.

## 2. Materials and Methods

### 2.1. Materials

Four kinds of steel were produced in this experiment. The chemical compositions are shown in Table 1. The main differences between the four steels are the concentrations of Nb and V. The production and rolling processes of the tested steels are as follows:

1. Preroll a 20 mm thick-plate sheet billet and heat to 1250°C for 2 h and then hot-roll to 3.4 mm, where the final rolling temperature was about 900°C
2. The cooling rate was set to approximately 45°C/s, and the hot billet was kept in the furnace at 620°C for 1 h, followed by air cooling
3. The oxide sheet and decarburization layer were polished
4. In the cold rolling process, the steel plate was heated to 900°C, isothermally insulated for 100 s, and then quenched in water
5. Finally, the steel was tempered at 200°C for 100 s and air-cooled to room temperature

### 2.2. Test Method

Optical microscopy (OM) analysis was performed along the rolling direction of the sample for mounting, grinding, polishing, and metallographic etching using 4% alcohol nitrate. The microstructural characterization using high-resolution electron backscattered diffraction (EBSD) was performed using an EDAX-TSL-OIM system with a step size of 100 nm. Transmission electron microscopy (TEM) analysis was performed on a JEOL 2100F at a working voltage of 200 kV, with energy dispersive X-ray spectrometers (EDS) by Oxford Instruments. To observe with TEM, thin foil specimens were prepared by wire cutting, mechanical polishing, and double-jet electropolishing (Denmark, Struers TenuPOL-5). The electropolishing solution was prepared by mixing 90% CH_3_COOH and 10% HClO_3_.

## 3. Results and Discussion

Figure 1 shows the metallographic analysis by OM of the experimental steels. Figures 1(a)–1(d) correspond to samples 1 to 4. The range is 160 × 160 mm of each sample. It can be seen in the figure that the materials are uniform martensitic structures. A comparison of these images shows that the microstructural density of each steel gradually increased from (a) sample 1 to (d) sample 4. Therefore, due to the addition of microalloying elements Nb and V, the microstructural refinement phenomenon is obvious. However, it is difficult to provide accurate and precise quantitative data to verify the PAGB or ML thickness.

Figures 2–5 present the EBSD analysis results within a 40 × 40 mm sample image. The figures show the results of the matrix structures, grain orientations, grain boundary (GB) rotation angles, and phase distribution, respectively.  Figure 2 is the EBSD image quality (IQ) mapping result. The PAGBs and very fine martensitic structures can be clearly observed. Two typical PAGBs are marked in Figure 2(a). It is speculated that the microstructure of the materials is refined after the addition of Nb or V. However, the grains in Figure 2(d) are much clearer and rather small.  Figure 3 shows the analytical results of the EBSD inverse pole figure (IPF). Obvious differences can be discerned between the grain orientations and morphology of the MLs. Most grains exhibit irregular orientation. Larger PAGBs are obvious in Figures 3(a) and 3(b). It is difficult to prove the locations of the PAGBs in Figures 3(c) and 3(d), as only very fine grains and martensite lath structures can be found.  Figure 4 shows the rotational angle analysis of the grain boundaries. A low angle grain boundary (LAGB) of 2-5° is marked in red, while a LAGB of 5-15° is marked in green. Rotational angles in the range of 15-180° are defined as high angle grain boundaries (HAGBs), as marked in blue. A careful comparison of Figures 3 and 4 shows that all PAGBs are HAGBs, while most of the very fine ML boundaries are considered to be LAGBs. The thickness of the common martensite lath is about 10-200 nm, while the minimum scanning beam size of EBSD is 100 nm. This may be the main reason why ML boundaries cannot be clearly identified.  Figure 5 shows the distribution of RA in martensitic steel by EBSD phase mapping. It can be seen from the figure that the RA (in green) in the material is dispersed in the material matrix. By comparing the locations of the grain boundaries, most of the RAs are near HAGBs. Image analysis results show that the contents of RA in samples 1 and 2 are around 0.7%, while those in samples 3 and 4 are around 1.4%.

Figure 6 shows the EBSD data analysis. The EDAX-TSL-OIM system of EBSD analysis gives the grain diameter of each grain. To clearly show the grain diameter distribution, each micron size range was counted.  Figure 6(a) shows that most of the diameters are less than 1 *μ*m in the four samples. In the 1–6 *μ*m range, the grain diameters of the four steels gradually decrease from sample 1 to sample 4. There were very few instances of the grain diameters exhibiting larger than 6 *μ*m in these samples. At the same time, the average grain diameter of the material can be obtained by the size statistics of all identifiable grains.  Figure 6(b) shows the average grain diameter of the four samples. Therefore, the EBSD grain diameter statistics clearly show progressive grain refinement from sample 1 to sample 4. The EBSD software can also provide the grain orientation angles and phase content.  Figure 6(c) shows the percentage of rotational angles of the grain boundaries. There were no specific change patterns found in the four samples.  Figure 6(d) presents the contents of the RA in the four samples. For samples 1 and 2, the content was near 0.7%, while in samples 3 and 4, the same value was approximately 1.4%.

In Figure 7, TEM was used to analyze the nanoprecipitated phase in the material, and energy dispersive X-ray spectrometry (EDS) was used to analyze the elemental composition alloy of the precipitated phase in the material. Sample 1 is Figure 7(a_1-3_), and sample 4 is Figure 7(b_1-3_). The composition test positions are marked on the figure, and the tables of the composition test results are shown on the map (Figures 7(a_2, 3_) and 7(b_2, 3_)). The concentrations of Nb, V, and Ti in the steel matrix were very low at position (Figure 7(a_2_)). The composition of the precipitated phase with a diameter of ~50 nm was measured at position (Figure 7(a_3_)). Results showed that the particles were enriched in Ti, while a small amount of Nb and V were also enriched. Two typical particles are selected in Figure 7(b_1_). The composition test results show that Ti particles with a size of ~20 nm are enriched in Nb and V, while particles of ~10 nm are enriched in Nb and only slightly enriched in Ti and V.

Nanoparticles, such as TiC, can nucleate and grow independently in martensitic steel [18, 20], and [24]. However, because of its high boundary energy, a larger amount of TiC is unfavorable for property improvement. Due to the addition of Nb and V, these elements were also precipitated near the TiC precipitation, resulting in the slow growth of TiC particles at this location. Compared with the analytical results of Figures 7(a_3_) and 7(b_3_), the size of the Nb-V-Ti particles (Figure 7(b_3_)) was smaller than that of normal TiC particles (Figure 7(a_3_)). However, it is worth noting that although the contents of Nb and V are very small in sample 1, their site of precipitation is still preferentially located near the TiC particles. When certain amounts of Nb and V are added, they can be nucleated by TiC (Figure 7(b_2_)) or independent nucleation (Figure 7(b_3_)).

Figure 8 shows closer observations of one precipitate at one location of Figure 7(b_3_).  Figure 8(a) shows the high-resolution TEM image, Figure 8(b) is the diffraction pattern from the yellow dotted square in Figure 8(a), Figure 8(c) is the high-resolution image after inverse Fourier transform, and Figure 8(d) is the interatomic distance measurement. The distance between atoms is 0.23 nm, which matches with the Nb_2_C (110) plane [39]. However, the analyzed carbides were mixed type (Ti, Nb, V,) C so that the lattice parameters do not correspond to those of pure species.

Figure 9 shows the bending and immersion test designed to verify the hydrogen embrittlement resistance of the material. After the sample was prepared into a thin sheet, drilling was carried out, and bending was completed using a hydraulic press on the tooling. All samples were cut and grounded at the same time. Then, the bolt was fixed, and all samples were simultaneously immersed in a sufficient amount of 0.5 mol/L hydrochloric acid solution that would cover the samples. A camera was used to record the breaking time of the four samples. It was found that the breaking times of the four samples were 2 h, 2.5 h, 7 h, and 9 h, respectively. All experimental conditions were the same, and as a result, it can be speculated that the reason for the difference is not due to preexisting cracks at the sample edge and the corrosion phenomena in the aggressive solution. It can be demonstrated that the addition of microalloying elements Nb and V refines the microstructure of the material, changes the content of RA, generates more nanoprecipitates, and creates many hydrogen traps. In conclusion, the addition of microalloying elements Nb and V significantly improves the hydrogen embrittlement resistance of the material.

It is believed that hydrogen possibly assembles near PAGBs, precipitates, and retained austenite.  Figure 10 shows the schematic diagram of the hydrogen distribution in high strength martensitic steel. These features have the potential to provide hydrogen embrittlement resistance by serving as hydrogen traps and limiting the availability of hydrogen to allow for embrittlement. By comprehensively comparing the above analysis, the addition of alloying elements V and Nb can play a role in grain refinement, where the Nb refinement effect is more obvious. Meanwhile, the addition of Nb (with or without V) clearly causes a larger amount of RA. With the addition of V, the composite of Nb-V-Ti-CN particles is smaller than the composite of Nb-Ti-CN particles, and the precipitation temperature is wider, which can effectively prevent the austenite grain growth and recrystallization process, and ultimately improves the strength and toughness of the material. Therefore, the addition of microalloying elements Nb and V significantly improves the hydrogen embrittlement resistance of the high strength martensitic steel.

## 4. Summary

In this paper, martensitic steels with the addition of different amounts of Nb and V are compared, where their effects near GBs and precipitate, and the retained austenitic characteristics of the steels on the hydrogen embrittlement resistance of high strength martensitic steels are analyzed. The test results showed that the addition of the microalloying elements Nb and V refines the microstructure of the material. The addition of Nb (with or without V) clearly causes a larger amount of RA. A large number of fine Nb-V-Ti compound nanoprecipitates are present in the material matrix, which creates many benign hydrogen traps. In conclusion, adding Nb and/or V can improve high strength martensitic steel and is an important direction for future applications.

## Figures and Tables

**Figure 1:** OM analysis of test steels, (a)–(d), respectively, corresponds to samples 1-4.

**Figure 2:** EBSD IQ analysis of samples 1–4.

**Figure 3:** EBSD IPF analysis of samples 1–4.

**Figure 4:** EBSD GB analysis of samples 1–4.

**Figure 5:** EBSD phases mapping analysis of samples 1–4.

**Figure 6:** EBSD data analysis on (a) diameter, (b) average diameter, (c) GBs, and (d) RA measurement.

**Figure 7:** TEM analyses of sample 1 (a_1_) and sample 4 (b_1_): (a_2_, a_3_, b_2_, and b_3_) EDS analyses on the respective marked positions, where the nested tables are the chemical compositions of each test.

**Figure 8:** Nanoprecipitate analysis by (a) high-resolution TEM imaging, (b) diffraction pattern from the yellow dotted square in (a), (c) high-resolution image after inverse Fourier transform, and (d) measurement of interatomic distance.

**Figure 9:** Diagram of bending and immersion experiments: (a) bending and (b) immersion test in 0.5 mol/L HCl solution. Images of (c) the tested sample as bending is fixed and (d) the tested sample after the immersion test with a fracture near the bending position.

**Figure 10:** Schematic diagram of hydrogen distribution in high strength martensitic steel.

**Table 1:** Chemical compositions of four kinds of tested steel (wt. %).

No.	C	Si	Mn	Cr	Cu	Ti	V	Nb
1#	0.23	0.22	1.2	0.2	0.01	0.03	0.001	0.003
2#	0.23	0.22	1.2	0.2	0.01	0.03	0.025	0.003
3#	0.23	0.22	1.2	0.2	0.01	0.03	0.001	0.035
4#	0.23	0.22	1.2	0.2	0.01	0.03	0.025	0.035

## Data Availability

No data were used to support this study.
